# The Bioinformatic Study Uncovers Probable Critical Genes Involved in the Pathophysiology of Biliary Atresia

This article has been retracted.

**DOI:** 10.1155/2022/9108804

**Published:** 2022-06-21

**Authors:** Si Chen, Songli Wu, Mingman Zhang

**Affiliations:** ^1^Children's Hospital of Chongqing Medical University, China; ^2^University-Town of Chongqing Medical University, China

## Abstract

**Background:**

Biliary atresia (BA) is an uncommon illness that causes the bile ducts outside and within the liver to become clogged in babies. If left untreated, the cholestasis causes increasing conjugated hyperbilirubinemia, cirrhosis, and hepatic failure. BA has a complicated aetiology, and the mechanisms that drive its development are unknown. The objective of this study was to show the role of probable critical genes involved in the pathophysiology of biliary atresia.

**Methods:**

We utilised the public Gene Expression Omnibus (GEO) microarray expression profiling dataset GSE46960 to find differentially expressed genes (DEGs) in 64 biliary atresia newborns, 14 infants with various causes of intrahepatic cholestasis, and 7 deceased-donor children as control subjects in our study. The relevant information was looked into. The important modules were identified after functional enrichment, GO and KEGG pathway analyses, protein-protein interaction (PPI) network analyses, and GSEA analysis.

**Results:**

The differential expression analysis revealed a total of 22 elevated genes. To further understand the biological activities of the DEGs, we run functional enrichment analyses on them. Meanwhile, KEGG analysis has revealed significant enrichment of pathways involved in activating cross-talking with inflammation and fibrosis in BA. SERPINE1, THBS1, CCL2, MMP7, CXCL8, EPCAM, VCAN, ITGA2, AREG, and HAS2, which may play a significant regulatory role in the pathogenesis of BA, were identified by PPI studies.

**Conclusion:**

Our findings suggested 10 hub genes and probable mechanisms of BA in the current study through bioinformatic analysis.

## 1. Introduction

Biliary atresia (BA) is a rare disease in which the bile ducts outside and inside the liver become blocked in newborns. Increasing evidence showed that newborn screening with direct or conjugated bilirubin results in earlier diagnosis. The serum bilirubin level after Kasai portoenterostomy is still the most accurate clinical predictor of native liver survival. Cholestasis causes increasing conjugated hyperbilirubinemia, cirrhosis, and hepatic failure if not treated [1, 2]. It is the most likely cause for a liver transplant in a youngster. BA has a tangled aetiology, with evidence pointing to viral, toxic, and genetic factors [3, 4]. The mechanisms that cause it are likewise unknown. We still do not know when BA starts or how to prevent the liver from deteriorating further [5]. A better knowledge of the aetiology of BA is required for novel therapy options other than liver transplantation to be developed. As a result, the goal of our research was to look at gene expression patterns in BA patients in order to look for potential biomarkers or pathological causes of the disease, as well as to find a better understanding and therapy for the condition.

## 2. Materials and Methods

### 2.1. Microarray Data

The gene expression profiling dataset GSE46960, which was deposited by Bessho et al. [6], was obtained using the Gene Expression Omnibus (GEO, https://www.ncbi.nlm.nih.gov/geo/) [7]. The dataset was created using the GPL6244 Affymetrix Human Gene 1.0 ST Array (transcript (gene) version) platform. Liver biopsy samples were obtained from 64 neonates with biliary atresia during an intraoperative cholangiogram, 14 age-matched babies with various kinds of intrahepatic cholestasis served as diseased controls, and 7 deceased-donor children served as normal controls. The age and sex of the participants, as well as their preoperative biochemical test data, were inaccessible because it was a public dataset, which looks to be a possible drawback. GPL6244's annotation file was also obtained from the GEO.

### 2.2. Differential Expression Analysis

Using the online analytic tool GEO2R, the expression profiles of BA, non-BA patients, and healthy controls were compared to find DEGs. *P* values and corrected *P* values were calculated using *T*-tests. The platform's gene probes were translated into gene names by referencing the GPL6244 platform. The genes in each sample were preserved if they matched two criteria: (1) a ∣log2 (fold − change) | >1 and (2) an adjusted *P* 0.05. We identified the most important genes when the DEGs were repeated. The DEGs were found by the intersection of the two datasets, which were conducted independently for the BA versus NC and BA vs. non-BA groups.

The online tool E Venn [8] (http://www.ehbio.com/test/venn/#/) was used to construct a Venn diagram of DEGs, and the heat map for the DEGs was made using the online tool xiantao Xue shu (https://www.xiantao.love/).

### 2.3. Functional Enrichment Analysis of DEGs

To improve the identification of the biological activities of DEGs, we used the web tool DAVID (https://david.ncifcrf.gov/) to conduct Gene Ontology (GO) terms [9] and Kyoto Encyclopedia of Genes and Genomes (KEGG) pathways [10]. Based on the GO analysis description, the gene function annotations were categorised as biological processes (BP), cellular components (CC), or molecular activities (MF). Statistical significance was defined as adjusted *P* values of less than 0.05. ClueGo [11, 12], a Cytoscape application (Cytoscape v3.8.0) plug-in, was utilised to demonstrate the relationship between gene enrichment analysis terms.

### 2.4. PPI Network Creation and Hub Gene Identification

A PPI network of DEGs was created using the Search Tool for the Retrieval of Interacting Genes (STRING11.5; https://string-db.org/). [13], with an interaction score cut-off of >0.4. The hub genes were found using Cytohubba [14], a Cytoscape software (Cytoscape v3.8.0) plug-in, and the key modules in the PPI network were found using molecular complex identification (MCODE 1.5.1) [15], another Cytoscape software plug-in. The DEG clustering and scoring parameters were MCODE score = 4, degree cut‐off = 2, node score cut‐off = 0.2, max depth = 100, and *k*‐score = 2.

### 2.5. GSEA Gene Set Enrichment Analysis

GSEA is a computer programme that determines if a set of genes that have been defined a priori demonstrate a statistically meaningful, congruent gap between different physiological situations (e.g., phenotypes). GSE46960 was submitted to Gene Set Enrichment Analysis with permutation = 1,000 using the GSEA tool (https://www.broadinstitute.org/gsea/) [16, 17]. A hypothetical *P* value was used to assess the statistically significant results of the enrichment score.

### 2.6. Statistical Analysis

Continuous normally distributed data are expressed as the means ± SDs. All statistical calculations were calculated through SPSS statistical software. *P* values < 0.05 were considered significant.

## 3. Results

### 3.1. Identification of DEGs in Biliary Atresia

The gene expression profile of the GSE46960 dataset comprised data from three separate groups (Table 1). Using a fold change (FC) value of (∣log2FC∣) > 2 and a *P* value of 0.05 as the cut-off, a total of 22 DEGs, all upregulated genes, were obtained from the notably regulated gene in the biliary atresia samples over both diseased control (non-BA) and normal control (NC) samples (Table 2). For the distribution of DEGs, an online tool was utilised to construct a Venn diagram and heat maps (Figures 1(a) and 1(b)).

### 3.2. GO and KEGG Pathway Analysis for Identifying the DEGs

DEGs were studied using the DAVID online tool for functional and pathway enrichment. The most three important processes revealed by GO analysis among the annotations of BP were extracellular matrix organization, cellular response to tumor necrosis factor, and cell adhesion. The three most important processes revealed among the CC annotations were extracellular space, extracellular area, and extracellular exosome. Finally, the three most significant processes among the MF annotations were receptor binding, glycosaminoglycan binding, and cytokine activity.  Table 3 and Figure 2 show the number of genes and *P* values of the top 8 enriched functional words based on the criteria.

The DEGs' cell signaling pathway enrichment study yielded a total of eight relevant pathways that were investigated. ECM-receptor interaction, malaria, the PI3K-Akt signaling pathway, and others were among the cellular signaling pathways linked to biliary atresia.  Table 4 and Figure 3 describe the specific enriched pathways discovered by DEG analysis.  Figure 4 shows the relationship between the words of gene enrichment analysis.

### 3.3. Construction of the PPI Network and Identification of Hub Genes

STRING (https://string-db.org/) is a public database that contains known and predicted protein interactions. PPI [18] is important for studying protein function since it can help elucidate the role of protein control. STRING's official website was used to submit the 22 DEGs from the GSE46960 dataset in order to get protein interrelationships. The minimum required interaction score was set at 0.15 in order to see the interaction networks with Cytoscape (version v3.9.0) [19]. There were 22 nodes and 107 edges in the PPI network that resulted. The network visualisation created using STRING's official website is shown in Figure 5(a). The degree of linkage between DEGs and genes was used to screen for hub genes, and the DEGs with the ten highest degrees were identified as hub genes (Table 5 and Figure 5(b)).

### 3.4. GSEA Analysis of All Detected Genes

GSEA was used to find gene sets with a statistically significant difference between BA and NC participants, and it revealed that the BA subjects had the highest enriched gene sets of all discovered genes. There are 4662 gene symbols in the dataset, 3651 of which are elevated in phenotype BA. ECM receptor interaction, integrin cell-surface interactions, and Andersen cholangiocarcinoma class1 were the top six most significant-enriched gene sets positively correlated with the BA subjects, followed by uterine fibroid up, ECM proteoglycans, and nonintegrin membrane ECM interactions (Figures 6(a)–6(f)).

## 4. Discussion

Biliary atresia (BA) is a fibroinflammatory disease of the intra- and extrahepatic biliary tree. In order to have a better understanding of the underlying cause(s) and pathogenesis of the disease, the National Institutes of Diabetes and Digestive and Kidney Diseases sponsored researches that study the promising and innovative approaches. In this investigation, we used the GEO database to screen for DEGs and acquire gene expression profiles from patients with BA, non-BA, and normal controls. There were a total of 22 DEGs confirmed.

The DEGs were considerably enriched in the cellular response to interleukin-1, according to BP in GO annotation, which was consistent with earlier evidence that inhibiting IL-1-mediated inflammation may be advantageous in selective liver fibrotic disease [20]. Other enhanced gene sets of DEGs in the BP of GO, such as immunological and inflammatory responses, have been linked to biliary atresia [21, 22]. The extracellular exosome was shown to be rich in CC.

Exosomes have been explored as disease biomarkers [23, 24] or cell-cell communication factors because of their role in carrying a variety of proteins, noncoding RNA, and coding RNA from different cells. A new study suggests that serum exosomal H19 might be exploited as a noninvasive diagnostic biomarker and treatment target for BA [25]. According to KEGG enrichment analysis, DEGs are also detected in the ECM-receptor interaction, focal adhesion, PI3K-Akt signaling pathway, and chemokine signaling pathway. All of these results corroborated previous findings that BA interacts with inflammation and fibrosis [26].

SERPINE1, THBS1, CCL2, MMP7, CXCL8, EPCAM, VCAN, ITGA2, AREG, and HAS2 were among the 10 hub genes discovered in this study. Interleukin- (IL-) 8 (CXCL8) may mediate liver damage in BA by enhancing ductular response and related hepatic fibrogenesis, according to Godbole et al. [27]. The serum MMP-7 test, according to Yang et al., shows excellent sensitivity and specificity for distinguishing BA from other newborn cholestasis and may be a valid biomarker for BA [28]. SERPINE1 can be targeted to prevent biliary fibrosis, according to Aseem et al.

The most significant-enriched gene set connected with the BA individuals, according to GSEA, was ECM receptor interaction. Many studies have linked oxidative stress to liver fibrosis. It has been discovered that ROS can activate KCs (Kupffer cells) to trigger the inflammatory response, which subsequently leads to HSC (activated hepatic stellate cells) activation to create ECM proteins [29, 30] and fibrosis. It will offer a fresh look at the treatment strategy for BA's fibrosis mechanism. The limit of this study is that there are only bioinformatic analysis and did not have cell and animal experiments. Therefore, many investigations need to be added to the article.

## 5. Conclusion

With bioinformatic analysis, we found 10 hub genes and probable mechanisms of BA in the current study. More research is needed to confirm the hub genes and identify relevant processes. All of the findings will pave the way for a possible treatment strategy for biliary atresia and associated fibrotic illnesses.

## Figures and Tables

**Figure 1:** (a) The selection of 22 genes based on BA vs. NC and non-BA as sick controls. (b) The expression data is displayed as a data matrix, with each row corresponding to a gene and each column to a sample. The colour ratio of the upper left corner is used to convey the amount of emotion. The top tree view demonstrates hierarchical clustering and indicates the degree of gene expression relatedness. Abbreviations: DEG: differentially expressed genes; BA: biliary atresia; non-BA: other causes of intrahepatic cholestasis except biliary atresia; NC: normal control; FC: fold change.

**Figure 2:** Results of GO enrichment. The ordinate shows the number and ratio of differentially expressed genes, whereas the abscissa reflects the enriched GO. Biological process, cellular component, and molecular function are all represented by distinct colours. Abbreviation: GO: gene ontology.

**Figure 3:** KEGG pathway analysis of the differentially expressed genes in BA. Abbreviations: KEGG: Kyoto Encyclopedia of Genes and Genomes; BA: biliary atresia.

**Figure 4:** Correlation between terms of gene enrichment analysis.

**Figure 5:** The PPI network and the most significant modules of DEGs. (a) String software was used to examine the PPI network. In the PPI network, there were 22 nodes and 120 edges. (b) CytoHubba found the most important module. Abbreviation: DEG: differentially expressed gene; PPI: protein-protein interaction.

**Figure 6:** GSEA plot showing the most enriched gene sets of all detected genes in the BA subjects. ECM receptor interaction (a), integrin cell surface contacts (b), and cholangiocarcinoma class1 are the top-six most significantly upregulated enriched gene sets in BA individuals (c). ECM proteoglycans (d), uterine fibroid uptake (e), nonintegrin membrane ECM interactions (f). Abbreviation: GSEA: gene set enrichment analysis; NES: normalized enrichment score.

**Table 1:** Details GEO biliary atresia data.

Sample	GEO	Platform	BA	Non-BA	NC
Liver	GSE46960	GPL6244	64	14	7

**Table 2:** List of genes specifically regulated in the biliary atresia samples over both diseased control (non-BA) and normal control (NC).

Gene symbol	Adjusted *P* value		Fold change		Description
	BA-NC	BA-non-BA	BA-NC	BA-non-BA	
Upregulated genes					
EPCAM	4.73E-25	4.56E-05	4.37	1.29	Epithelial cell adhesion molecule
SPP1	8.86E-17	4.56E-05	3.26	1.37	Secreted phosphoprotein 1
ANKRD1	4.14E-10	1.73E-06	3.11	2.05	Ankyrin repeat domain 1
MMP7	3.76E-08	8.21E-05	2.94	1.85	Matrix metallopeptidase 7
LUM	3.21E-12	6.17E-05	2.70	1.26	Lumican
RGS4	7.25E-12	5.86E-04	2.54	1.03	Regulator of G-protein signaling 4
EMP1	1.16E-05	1.96E-03	2.40	1.41	Epithelial membrane protein 1
CFTR	1.41E-08	2.82E-03	2.33	1.05	Cystic fibrosis transmembrane conductance regulator
HAS2	3.69E-06	1.62E-04	2.28	1.56	Hyaluronan synthase 2
KRT23	1.34E-08	5.29E-04	2.19	1.14	Keratin 23
VCAN	6.40E-10	1.52E-05	2.12	1.32	Versican
CXCL8	3.55E-09	4.56E-05	1.93	1.20	C-X-C motif chemokine ligand 8
CCL20	1.75E-03	1.14E-02	1.87	1.24	C-C motif chemokine ligand 20
VTCN1	4.14E-08	1.11E-04	1.81	1.09	V-set domain containing T cell activation inhibitor 1
ITGA2	6.29E-07	1.50E-04	1.68	1.10	Integrin subunit alpha 2
SERPINE1	1.28E-02	9.47E-03	1.53	1.36	Serpin family E member 1
THBS1	5.61E-06	3.54E-04	1.52	1.00	Thrombospondin 1
CCL2	2.51E-04	4.05E-05	1.38	1.37	C-C motif chemokine ligand 2
TM4SF1	1.14E-03	1.52E-05	1.38	1.71	Transmembrane 4 L six family member 1
LAMC2	1.99E-06	4.56E-05	1.35	1.02	Laminin subunit gamma 2
AREG	6.89E-03	2.44E-03	1.34	1.28	Amphiregulin
SLC2A3	1.05E-02	2.66E-03	1.15	1.16	Solute carrier family 2 member 3

**Table 3:** Top 8 of the most significantly enriched GO terms.

Pathway ID	Terms	Gene count	*P* value
BP			
GO:0030198	Extracellular matrix organization	7	5.60E-08
GO:0071356	Cellular response to tumor necrosis factor	6	1.19E-07
GO:0071347	Cellular response to interleukin-1	5	1.08E-06
GO:0071222	Cellular response to lipopolysaccharide	5	6.97E-06
GO:0007155	Cell adhesion	6	1.26E-04
GO:0006954	Inflammatory response	5	7.57E-04
GO:0008284	Positive regulation of cell proliferation	5	1.63E-03
GO:0006955	Immune response	4	1.12E-02
CC			
GO:0005615	Extracellular space	11	7.80E-07
GO:0005576	Extracellular region	10	3.53E-05
GO:0009986	Cell surface	6	3.13E-04
GO:0031012	Extracellular matrix	5	3.28E-04
GO:0009897	External side of plasma membrane	3	2.47E-02
GO:0070062	Extracellular exosome	8	3.29E-02
GO:0048471	Perinuclear region of cytoplasm	4	3.32E-02
GO:0005578	Proteinaceous extracellular matrix	3	3.77E-02
MF			
GO:0005539	Glycosaminoglycan binding	5	9.29E-05
GO:0005125	Cytokine activity	5	1.20E-04
GO:0005102	Receptor binding	9	1.51E-04
GO:0008201	Heparin binding	4	8.46E-04
GO:0008009	Chemokine activity	3	1.52E-03
GO:1901681	Sulfur compound binding	4	2.49E-03
GO:0043236	Laminin-binding	2	2.92E-02
GO:0050840	Extracellular matrix binding	2	3.04E-02

Notes. GO: Gene Ontology; BP: biological progress; CC: cellular component; MF: molecular function.

**Table 4:** Significantly enriched KEGG pathway.

Pathway ID	Term	Gene count	*P* value	Genes
hsa04512	ECM-receptor interaction	4	5.10E-04	THBS1, ITGA2, LAMC2, SPP1
hsa05144	Malaria	3	3.69E-03	CCL2, THBS1, CXCL8
hsa04510	Focal adhesion	4	6.06E-03	THBS1, ITGA2, LAMC2, SPP1
hsa05323	Rheumatoid arthritis	3	1.15E-02	CCL20, CCL2, CXCL8
hsa05142	Chagas disease (American trypanosomiasis)	3	1.58E-02	CCL2, CXCL8, SERPINE1
hsa04151	PI3K-Akt signaling pathway	4	2.46E-02	THBS1, ITGA2, LAMC2, SPP1
hsa04062	Chemokine signaling pathway	3	4.66E-02	CCL20, CCL2, CXCL8

Notes. KEGG: Kyoto Encyclopedia of Genes and Genomes.

**Table 5:** Top 10 hub genes ranked by Cytobubba.

Gene symbol	Score	Full name	Distribution
SERPINE1	32	Serpin family E member 1	Serine protease inhibitor; plasminogen activator inhibitor 1. Tissue plasminogen activator, urokinase, protein C, and matriptase-3/TMPRSS7 are all attracted to this inhibitor. Its quick interaction with PLAT might be a crucial control point in fibrinolysis regulation.
THBS1	32	Thrombospondin 1	Cell-to-cell and cell-to-matrix adhesion glycoprotein thrombospondin-1 modulates cell-to-cell and cell-to-matrix connections. This chemical binds to heparin. Dentin and dental pulp dentinogenesis and/or maintenance may be affected (by similarity). A CD36 ligand is responsible for the antiangiogenic actions. It has a function in the ER stress response by interacting with the activating transcription factor 6 alpha (ATF6), which produces adaptive ER stress response factors (by similarity)
CCL2	30	C-C motif chemokine ligand 2	Chemotactic factor with a C-C motif, which attracts monocytes and basophils but not neutrophils or eosinophils. Increases the antitumor activity of monocytes. Has been linked to the development of disorders with monocytic infiltrates, such as psoriasis, rheumatoid arthritis, and atherosclerosis. During the disease process of atherosclerosis, it may be implicated in the recruitment of monocytes into the artery wall.
MMP7	30	Matrix metallopeptidase 7	Matrilysin degrades casein, gelatins of types I, III, IV, and V, and fibronectin. Activates procollagenase; M10 matrix metallopeptidases
CXCL8	30	C-X-C motif chemokine ligand 8	IL-8 is a chemotactic factor that attracts neutrophils, basophils, and T cells but not monocytes. It has a role in neutrophil activation as well. In response to an inflammatory stimulation, it is secreted by a variety of cell types. When compared to IL-8 (1-77), IL-8 (6-77) has a 5-10-fold higher activity on neutrophil activation, IL-8 (5-77) has enhanced activity on neutrophil activation, and IL-8 (7-77) has a stronger affinity to CXCR1 and CXCR2 receptors.
EPCAM	28	Epithelial cell adhesion molecule	Intestinal epithelial cells (IECs) and intraepithelial lymphocytes (IELs) establish a physical homophilic contact molecule at the mucosal epithelium to build an immunological barrier as a first line of defence against mucosal infection. Plays a function in the proliferation and differentiation of embryonic stem cells. The expression of FABP5, MYC, and cyclins A and E is all increased.
VCAN	24	Versican	Intercellular signaling and cell-extracellular matrix interactions may be mediated by the Versican core protein. It might play a part in cell motility, proliferation, and differentiation. Has a C-type lectin domain that binds hyaluronic acid.
ITGA2	24	Integrin subunit alpha 2	Integrin alpha-2 (integrin alpha-2/beta-1) is a receptor for laminin, collagen, collagen C-propeptides, fibronectin, and E-cadherin. It recognises the proline-hydroxylated sequence G-F-P-G-E-R in collagen. Platelet and other cell adhesion to collagens, collagen and collagenase gene expression control, force creation, and structuring of newly formed extracellular matrix are all mediated by CD molecules.
AREG	24	Amphiregulin	Amphiregulin is a ligand for the EGF receptor/EGFR. Amphiregulin is an amitogen and autocrine growth factor for a range of target cells, including astrocytes, Schwann cells, and fibroblasts.
HAS2	22	Hyaluronan synthase 2	Hyaluronan synthase 2 adds GlcNAc or GlcUA monosaccharides to the nascent hyaluronan polymer. As a result, it is essential for the formation of hyaluronan, a major component of most extracellular matrices that regulates cell adhesion, migration, and differentiation and plays a structural role in tissue architecture. This is one of the isozymes that catalyses the process and is responsible for the production of high-molecular-mass hyaluronan. A key phase in the creation of the heart is the conversion of endocardial cushion cells to mesenchymal cells.

## Data Availability

The data could be obtained from contacting the corresponding author.
